The article "Loperamide-Induced Cardiac Events: Case Reports and Review" was published in 2021. Journal: Cureus.

# Loperamide-Induced Cardiac Events: Case Reports and Review

**DOI:** 10.7759/cureus.20744

**Published:** 2021-12-27

**Authors:** Vivek Modi, Matthew Krinock, Ravi Desai, Steven Stevens, Sudip Nanda

**Affiliations:** 1 Cardiology, St. Luke’s University Health Network, Bethlehem, USA; 2 Cardiology, Lehigh Valley Heart and Vascular Institute, Allentown, USA; 3 Electrophysiology, St. Luke’s University Health Network, Bethlehem, USA

**Keywords:** brugada ecg pattern, opioid, clinical case report, qt interval prolongation, loperamide cardiotoxicity

## Abstract

Reports of cardiac arrhythmia secondary to loperamide toxicity have become increasingly common in the literature. We present two patients in their mid-20s, each having overdosed on loperamide and subsequently manifesting life-threatening cardiac arrhythmias not otherwise explained by known pathology. An analysis of the limited research available indicates that loperamide’s capacity to block ion channels may be responsible for these events. A better mechanistic understanding of loperamide’s effects can help inform clinical management of patients with these life-threatening symptoms as at this time no set guidelines for management have yet been established.

## Introduction

The use of loperamide for self-managing opioid addiction is becoming an increasingly prevalent public health concern. Despite its benign use for gastrointestinal complaints, excessive loperamide consumption has been associated with lethal cardiac arrhythmias. Although awareness has increased, cases of toxicity present a challenging diagnosis for physicians as no standardized management is established. As of now, the best practice hinges on an index of suspicion on behalf of electrophysiologists and physicians on the frontlines of the opioid epidemic. We present two cases of loperamide overdose, highlighting the variability in presentation and evaluating the evidence for effective management of similar patients.

## Case presentation

Patient one

The patient was a 28-year-old male with a past medical history of previous heroin abuse. He started taking loperamide to help his withdrawal symptoms, consuming at least 100 capsules (200 mg) of loperamide daily for an estimated six months prior to presentation.

Two days prior to presentation at the hospital, he reported feeling generalized weakness, difficulty taking deep breaths, and mild lightheadedness. Upon arrival at the hospital, he was found to have an abnormal electrocardiogram (EKG) with a widened QRS and prolonged QT interval. He was given 4 amps of sodium bicarbonate, improving his abnormal intervals. He was then started on a bicarbonate drip and admitted to the medical intensive care unit for further observation. A day after the bicarbonate drip was turned off, he developed an episode of polymorphic ventricular tachycardia. He was then restarted on the bicarbonate drip with the addition of an isoproterenol infusion to control his developing torsades de pointes. Subsequently, he was given a temporary pacemaker and was V paced for eight days at 90/minute. He was then discharged and enrolled himself in a substance abuse rehabilitation program. Figure 1 shows the patient’s EKGs.

**Figure 1:** EKGs of patient one EKG: electrocardiogram

Patient two 

The patient was a 26-year-old female with a prior history of heroin abuse, depression, and anxiety who presented to the hospital complaining of recurrent episodes of near syncope, palpitations, and fatigue. She reported five episodes within the previous two months, describing the sensation as “feeling shaky and legs giving away.” She regularly took amphetamine/dextroamphetamine, clonazepam, levothyroxine, and, within the last four months, metoprolol. At the onset of her symptoms, she had begun to take roughly 200 mg loperamide daily. She denied having used heroin since September 2015 and had not received methadone treatment recently.

On presentation, her urine contained traces of amphetamines. Her EKG was abnormal with a Brugada type 1 pattern, right bundle branch block, first-degree AV block, 122 ms widened QRS, and a QT prolongation of greater than 600 ms. Telemetry showed sinus bradycardia at 50-60 beats/minute without concurrent tachyarrhythmia. Figure 2 shows the patient’s EKG.

**Figure 2:** EKG of patient two EKG: electrocardiogram

Table 1 shows a comparison of the presentation and symptoms of patient one and patient two.

**Table 1:** Comparison of patient one and patient two

Patient one	Patient two
200 mg/six months	200 mg/two months
Wide QRS and QT interval prolongation	Wide QRS and QT interval prolongation
Ventricular tachycardia	Brugada type 1
Torsades de pointes	Right bundle branch block
	First-degree AV block
	Sinus bradycardia

## Discussion

Loperamide hydrochloride is a diphenylmethane piperidine compound marketed to control diarrhea, inflammatory bowel disease, and gastroenteritis. As a mu opioid receptor agonist, its action at therapeutic doses is primarily confined to the myenteric plexus of the enteric nervous system, resulting in slowed transit time [1-4]. Loperamide’s interaction with the mu opioid receptor is depicted in Figure 3.

**Figure 3:** Loperamide binding activates mu opioid receptor, relaxing the intestines and decreasing gastric motility

When appropriately dosed, loperamide’s actions are localized to the bowel due to low oral bioavailability (0.3%) and significant first-pass metabolism by hepatic CYP3A4, CYP3C8, and P-glycoprotein. Per these limitations, murine models suggest a lethal dose of 105 mg/kg, whereas the recommended dose is 16 mg/day [1,4]. Nonetheless, mounting anecdotal evidence of loperamide’s toxicity prompted the Food and Drug Administration (FDA) to release a warning statement for physicians in July 2016 to maintain a high index of suspicion in at-risk patients [1,5].

Loperamide toxicology

Due to its activity at opioid receptors, loperamide has been called the “poor man’s methadone,” an inexpensive means to soften street and prescription opioid withdrawal. Knowledge of this off-label use spread over the Internet [1,6]. Individuals appreciating the opioid effects may present with plasma levels greater than 1,000 times the recommended concentrations [1,5]. Case reports have been reported of patients presenting with abnormal symptoms after substantial doses of loperamide, mirroring the effects of harder opioid overdoses, such as heroin [1,2,7-9]. Recently, the FDA began compiling cases of presumed loperamide toxicity, citing 48 loperamide cardiac cases since the drug’s approval in 1976 with half of the cases appearing in the year 2010 alone. However, because loperamide is not commonly ordered in toxicological screens, there are likely many overlooked cases [1]. Table 2 provides a review of reported loperamide toxicity [1-3,5].

**Table 2:** FDA-reported cardiac cases associated with loperamide use FDA: Food and Drug Administration

Cardiac-related events	Numbers reported to the FDA or assessed in the literature
Syncope	24
Cardiac arrest	13
QT interval > ~450 ms	13
Ventricular tachycardia, broad complex tachycardia	10
Torsades de pointes	10
Death	3
Brugada syndrome type 1 EKG (ST elevation in V1-V3, right bundle branch block)	1

Pharmacology

In the reported cases of loperamide toxicity, in descending order of frequency, the cardiac events were as follows: syncope, cardiac arrest, QT interval prolongation, ventricular tachycardia, torsades de pointes, and Brugada pattern [1,5]. Because these findings of QT prolongation, torsades de pointes, and Brugada pattern are known to be caused by well-studied electrolyte imbalances or channel dysfunctions, a closer evaluation of loperamide’s pharmacologic actions is warranted.

Two small studies performed on rodent brains indicate a substantial decrease in in vitro calcium release post-high-dose administration of loperamide, specifically indicating nonselective high-voltage calcium channel antagonism [1,2,10,11]. Additional studies suggest that elevated doses can also inhibit N-methyl-D-aspartate (NMDA) receptors, calmodulin, delayed rectifier potassium channels, and perhaps voltage-gated sodium channels, although this last example has not been rigorously confirmed [2-4,12,13]. Suprathreshold doses are necessary to interact with these extra-gastrointestinal channels [2,4,5,14]. Frequent excessive dosing has been shown to cause bioaccumulation of loperamide in fat deposits, which can lead to supratherapeutic tissue drug concentrations [3-5,8]. Figure 4 shows the proposed action potential changes from opioid toxicity.

**Figure 4:** Role of delayed rectifier potassium channels and voltage-gated calcium channels in the cardiac action potential. Loperamide can block calcium and potassium channels. Calcium channel blockade elongates phase 0 and 4 of the cardiac action potential. Potassium channel blockade delays phase 3. Both of these effects can lengthen action potential and increase susceptibility to arrhythmias

The successful management of patient one with sodium bicarbonate, which is known to reverse sodium channel blockade, supports the sodium channel blockade hypothesis, although currently there is no research evidence of the same. Blockade of potassium and calcium channels explains widening QTc, bradycardia, and AV block [6].

Treatment approaches

Acute Medical Management

The first step in managing suspected loperamide toxicity is to recognize and respond to life-threatening arrhythmias. Drug screening has limited efficacy. Loperamide’s tendency to accumulate in fat may lead to apparently therapeutic plasma levels in the presence of toxic symptoms. While these patients can be identified by multiday persistence of therapeutic concentration despite abstinence, few patients will be hospitalized long enough to trend this finding [3,8].

Anti-arrhythmics have had limited success in loperamide toxicity [7,15]. Isoproterenol has been used successfully in toxicity, including in patient one, with Brugada pattern, bradycardia, torsades de pointes, and ventricular arrhythmias [8]. Bicarbonate use has been successful for some and not for others [2,15]. Potassium and magnesium should be aggressively repleted to prevent worsening QT prolongation [8]. For unstable patients, electrical overdrive pacing should be considered [15,16]. Acute overdose warrants activated charcoal with at least one recommendation allowing for an extended period of administration due to the lack of other treatment options as well as the known effects on peristalsis [3]. Additional anecdotal evidence also suggests a role for lipid emulsion therapy including lipid heavy parenteral nutrition [3]. This acts as a “lipid sink,” reducing loperamide accumulation in the adipose tissue [10,17]. If loperamide abuse secondary to opioid withdrawal or addiction is suspected, the patient should be referred to the proper drug abuse clinic for treatment. Table 3 lists various treatment approaches tried for loperamide toxicity in literature, along with its characteristics [2,3,15,18-20].

**Table 3:** Therapies used in literature ILE: intravascular lipid emulsion

Treatment	Mechanism of action	Dose	Advantages	Disadvantages	Successes	Failures
Anti-arrhythmic drugs	Pharmacological attenuation of arrhythmia	Depends on agent	Well studied with known effects	Drug-induced arrhythmia	None	Marraffa et al. [15], Enakpene et al. [2]
Sodium bicarbonate	Reversal of Na­^+^ blockade	1 mg/kg loading followed by 0.5 mg/kg every 10 minutes as needed	Increased survival in arrhythmia	Aggressive treatment can cause metabolic alkalosis and hypokalemia		Enakpene et al. [2], Marraffa et. al. [15]
Isoproterenol	Sympathomimetic action	1.25 mL/minute followed by 2–20 mL/minute as needed	Rapid onset of action	Can cause drug-induced arrhythmia and cardiovascular collapse	Vaughn et al. [18], Marraffa et al. [15], Enakpene et al. [2], Spinner et al. [20], Eggleston et al. [19]	
Transvenous pacing	Overdrive pacing		Safe and low-risk procedure	Requires skill and equipment for placement	Vaughn et al. [18], Marraffa et al. [15], Spinner et al. [20], Eggleston et al. [19]	
Lipid emulsion therapy	Hydrophobic lipid “sink” for toxin	1.5 mL/kg of 20% ILE followed by 0.25 mg/kg/minute	Promising results in general drug toxicity management	Protocols are not standardized		Enakpene et al. [2], Marraffa et al. [15]

## Conclusions

The use of loperamide as an opioid substitute presents a novel but pressing challenge for medical teams. As there is currently no pharmacologic mechanism explaining the observed arrhythmias, no treatment protocol has yet been established for these patients. Until such a time as there is better research supporting the appropriate management of these patients, physicians must rely on clinical savvy and anecdotal successes, although the latter presents frequently conflicting evidence. Appropriate prevention and awareness on behalf of medical professionals and the community at large are also necessary to identify and circumvent the potential consequences of this form of self-medication.
